# MicroRNA-140-5p inhibits cell proliferation, migration and promotes cell apoptosis in gastric cancer through the negative regulation of THY1-mediated Notch signaling

This article has been retracted.

**DOI:** 10.1042/BSR20181434

**Published:** 2019-07-23

**Authors:** Kun Wu, Jun Zou, Chao Lin, Zhi-Gang Jie

**Affiliations:** 1 Medical College of Nanchang University, Nanchang 330006, P.R. China; 2 Department of Surgery, Jiangxi Tumor Hospital, Nanchang 330029, P.R. China; 3 Department of Surgery, The First Affiliated Hospital of Nanchang University, Nanchang 330006, P.R. China

**Keywords:** Gastric cancer, microRNA-140-5p, Migration, Notch signaling pathway, Proliferation, THY1

## Abstract

Studies have highlighted the importance of microRNAs (miRs) in the development of various cancers, including gastric cancer (GC), a commonly occurring malignancy, accompanied by high recurrence and metastasis rate. The aim of the current study was to investigate the role of miR-140-5p in GC. Microarray expression profiles were initially employed to screen the differentially expressed gene related to GC, and the miR regulating the gene was predicted accordingly. The data obtained indicated that thymus cell antigen 1 (*THY1*) was differentially expressed in GC and confirmed to be a target gene of miR-140-5p. Poorly expressed miR-140-5p and highly expressed *THY1* were observed in the GC tissues. SGC-7901 cells were treated with miR-140-5p mimic/inhibitor, siRNA against *THY1* and siRNA against *Notch1* in order to determine their regulatory roles in GC cell activities. The relationship of miR-140-5p, *THY1* and the Notch signaling pathway was subsequently identified. Moreover, cell proliferation, migration, invasion and apoptosis were determined using 3-(4,5-dimethylthiazol-2-yl)-5(3-carboxymethonyphenol)-2-(4-sulfophenyl)-2H-tetrazolium (MTS), wound-healing, transwell assay and flow cytometry, respectively. The overexpression of miR-140-5p and silencing of *THY1* resulted in a diminished expression of the Notch signaling pathway-related proteins, as well as inhibited proliferation, migration and invasion of GC cells, enhanced expression of pro-apoptotic proteins in addition to elevated apoptosis rate. Taken together, the present study suggests that miR-140-5p directly targets and negatively regulates *THY1* expression and inhibits activation of the Notch signaling pathway, whereby the up-regulation of miR-140-5p inhibits development of GC, highlighting the promise of miR-140-5p as a potential target for GC treatment.

## Introduction

Gastric cancer (GC) ranks as the fourth most prevalent cancer malignancy as well as the second most common cause of cancer-related mortality worldwide [1]. GC diagnosis is often accompanied by a poor prognosis, with patients in China often diagnosed at a late stage of the disease [2]. In approximately 90% of all cancer cases, death is often the general outcome with invasion and metastasis the prime causes [3]. Metastatic GC represents a life-threatening condition linked with poor overall patient survival rates, which underlines an urgent and crucial need for effective novel treatment options [4]. Although recent studies have explored various molecular targets for the diagnosis and treatment of GC, relatively few targets have been developed and approved as tools capable of clinically improving the treatment outcomes of metastatic GC patients [5]. A growing number of studies have emphasized the association of microRNA (miRs) with the pathogenesis of cancer in addition to various genetic alterations [6]. Various miRs have been reported to play a crucial role in the regulation of a large array of gene post-transcriptional processes, with studies implicating them in other cellular process such as cell growth, development, differentiation, proliferation and apoptosis [7]. A similar mechanism of expression has been linked with a large number of cellular genes, with the expression of miRs shown to be regulated by transcription factor binding, genetic and epigenetic alterations as well as chromosomal rearrangements [8,9].

Thymus cell antigen 1 (*THY1*) is a key regulator involved in the cellular interactions between a cell and its matrix [10]. A previous study indicated that *THY1*, also known as the *CD90* gene, exhibits a high expression level in GC while acting to inhibit the apoptosis of GC cells by regulating the expression of the secreted protein acidic and rich in cysteine (SPARC) protein [11]. Bioinformatics online prediction software as well as the application of a dual luciferase reporter gene assay in this study provided evidence confirming *THY1* as a direct target gene of miR-140-5p. Studies have indicated that miR-140-5p acts as a tumor suppressor in colorectal cancer, carcinoma of the bile duct and hypopharyngeal carcinoma [12–14]. Moreover, the down-regulated expression of miR-140-5p has been observed in GC with reports suggesting it could act to inhibit gastric cell proliferation [15]. Also, *THY1* can negatively regulate RhoA [16], with a previous study suggesting that RhoA regulates the Notch signaling pathway [17]. The Notch pathway is one of the key pathways related to stem cell biology and cancers [18]. Targeting Notch inhibits tumor growth and moderates the apoptosis of tumor initiating cells [19]. Previous studies have revealed activation of the Notch signaling pathway in GC cells along while linking it with the process of tumor formation and development [20]. An accumulating amount of evidence has highlighted the ability of *THY1* to regulate the Notch signaling pathway, while a lack of investigation into the relationship between miR-140-5p, *THY1* and Notch signaling pathway has been conducted. Hence, the current study was performed with the aim of investigating the mechanism by which miR-140 influences GC cell proliferation.

## Materials and methods

### Differential analysis of genes in GC

Gene Expression Omnibus (GEO) database (https://www.ncbi.nlm.nih.gov/geo/) was explored in order to obtain the microarrays related to GC. Limma package was employed for the differential analysis of GC expression chips, with |log foldchange (FC)| > 2 and *P*-value <0.05 serving as the screening criteria for the differentially expressed genes. The ‘pheatmap’ package was used to construct the expression heatmap of the differentially expressed genes.

### Gene retrieval and interaction analysis of GC

MalaCards database (http://www.malacards.org/) was explored in order to detect genes related to GC, while the STRING database (https://string-db.org/) was employed for correlation analysis between the differentially expressed genes and GC-related genes. Besides, the gene interaction network diagram was plotted using the Cytoscape software.

### Prediction of miR regulating *THY1*

MirDIP database (http://ophid.utoronto.ca/mirDIP/index.jsp#r) and miRGator database (http://mirgator.kobic.re.kr/) were used to predict the miRs regulating *THY1*, and the intersection of the forecast results was determined.

### Study subjects

A total of 105 patients, consisting of 67 males and 38 females, whose GC diagnosis had been confirmed by the Oncology Department of The First Affiliated Hospital of Nanchang University between January 2014 and January 2017, were recruited for the purposes of the study [21]. All patients’ cancer tissues and corresponding paracancerous tissues were confirmed and collected accordingly. The age range of the patients was between 34–72 years, with an average age of 53.2 ± 5.9 years. All enrolled patients were yet to receive any chemotherapy or radiotherapy prior to the operation, and classified according to the World Health Organization (WHO) histologic classification standard of GC [22], with 27 cases confirmed to be highly differentiated, 34 cases of middle differentiation, 44 cases of low differentiation, 60 cases with lymphatic metastasis, 45 cases with no metastasis, 9 cases at stage I, 18 cases at stage II, 47 cases at stage III, 31 cases at IV stage, 46 cases with an unaffected serosa and 59 cases with serosal invasion.

### Cell culture

Normal gastric epithelial cells (GES-1) and GC cell lines (MKN-28, MGC-803, SGC-7901, AGS and MKN-45) were purchased from American Type Culture Collection (ATCC, Manassas, VA, U.S.A.). The cells were cultured in Roswell Park Memorial Institute (RPMI) 1640 medium (31800-022, HyClone, UT, U.S.A.) containing 10% inactivated fetal bovine serum (FBS; 16000-044, Gibco Company, Grand Island, NY, U.S.A.) and 100 units/ml penicillin-streptomycin (15140122, Company, Grand Island, NY, U.S.A.) in a 5% CO_2_ incubator (3110 water jacket series, Thermo Fisher Scientific Inc., Waltham, MA, U.S.A.) at 37°C. The expression of miR-140-5p was subsequently determined through the application of reverse-transcription quantitative polymerase chain reaction (RT-qPCR), and the cell line with the lowest miR-140-5p expression versus that of GES-1 cells was selected for subsequent experiments, and another cell line (MGC-803) was selected for verification of the results. The following experiments were conducted after cell digestion with 0.25% trypsin (25200-056, Gibco Company, Grand Island, NY, U.S.A.) with 80% cell coverage confirmed under a microscopic view.

### Cell transfection and grouping

Oligonucleotide fragments miR-140-5p mimic, negative control (NC) (NC oligo-nucleotides) miR-140-5p inhibitor, si-NC and si-*THY1* were all purchased from Shanghai GenePharma Co., Ltd. (Shanghai, China). The cells were subsequently transfected and assigned into the control, NC, miR-140-5p mimic, miR-140-5p inhibitor, si-NC, si-*THY1* miR-140-5p inhibitor + si-*THY1*, and miR-140-5p inhibitor + si-*Notch1* groups. The wild-type (wt) sequence of *THY1* was 5′-CCUGACUUCUCCCCAA***CCA***CUU-3′ and mutant (mut) sequence was 5′-CCUGACUUCUCCCCAA***UUG***CUU-3′, which were synthesized by Shanghai GenePharma Co., Ltd. (Shanghai, China). The sequence of *Notch1*-specific siRNA (Santa Cruz Biotechnology, Santa Cruz, CA, U.S.A.) was 5′-GAT CCA GGA AGA GTG TTC CTG ATT TTC AAG A-3′. The cells were inoculated in a plate and incubated under conventional conditions 24 h prior to transfection. The culture medium was renewed 1 h prior to the transfection, followed by the addition of 2 ml of conventional culture medium per well. The mixture for transfection was prepared in accordance with the instructions of the Lipofectamine 2000 kit (11668-027, Invitrogen Inc., Carlsbad, CA, U.S.A.). Serum- and penicillin/streptomycin-free medium was added to the control group. Serum- and penicillin/streptomycin-free medium containing the corresponding oligonucleotide fragments (the final concentration was 300 pmol/well) covered by liposome (Invitrogen Inc., Carlsbad, CA, U.S.A.) was added to the corresponding groups. The transfected cells were then blocked with serum-free medium over a period of 4 h, followed by a further incubation with 5% CO_2_ at 37°C with 10% FBS.

### Dual-luciferase reporter gene assay

Online bioinformatics prediction software microrna.org was employed in order to predict the binding sites of miR-140-5p and *THY1*. A *THY1* 3′-untranslated region (UTR) fragment with or without miR-140-5p binding sites was inserted into pMIR-REPORT vectors (Ambion, Carlsbad, CA, U.S.A.). The wt plasmid pMIR-*THY1*-3′-UTR-wt (*THY1*-wt) and the mutant pMIR-*THY1*-3′-UTR-mut (*THY1*-mut) were constructed. The wt sequence of *THY1* was 5′-CCUGACUUCUCCCCAA***CCA***CUU-3′ and mut sequence was 5′-CCUGACUUCUCCCCAA***UUG***CUU-3′. HEK 293T cells were inoculated in a 96-well plate at a density of 4 × 10^4^ cells/well 24 h before transfection, with four duplicated wells set up. The culture medium was renewed 1 h before transfection and each well was added with the conventional culture medium. The transfection mixture was prepared in accordance with the instructions of the Lipofectamine 2000 kit (11668-027, Invitrogen Inc., Carlsbad, CA, U.S.A.) and introduced into the plate after discarding the culture medium. A dual-luciferase reporter gene assay kit (Promega Corporation, Madison, WI, U.S.A.) was employed in order to detect transcriptional activity 24 h after transfection. The co-transfection groups were as follows: miR-140-5p mimic + *THY1*-wt, NC + *THY1*-wt, NC + *THY1*-mut, miR-140-5p mimic + *THY1*-mut. All experiments were performed in triplicates.

### RT-qPCR

Total RNA was extracted from the cancer tissues, paracancerous tissues and cells in each group using TRIzol (15596026, Invitrogen Inc., Carlsbad, CA, U.S.A.) in accordance with the instructions of the miRNeasy Mini kit (217004, Qiagen Company, Hilden, Germany). The concentration and purity of the extracted RNA was detected using NanoDrop2000 (NanoDrop 2000c, Thermo, NY, U.S.A.). The collected RNAs were preserved at −80°C. The special stem ring RT primer (0.15 µM) was used to synthesize cDNA of miR-140-5p and small nuclear RNA U6 (U6) (Table 1). The PCR primers were designed using the Primer5.0 based on the gene sequences from the Genbank, and synthesized by Shanghai GenePharma Co., Ltd. (Shanghai, China) (Table 1). ABI PRISM 7500 real-time PCR System (ABI Company, Oyster Bay, NY, U.S.A.) and SYBR Green I Luciferase Kit (DRR041A, Takara Holdings Inc., Kyoto, Japan) were adopted for the PCR. U6 and glyceraldehyde-3-phosphate dehydrogenase (GAPDH) were regarded as the internal controls for miR-140-5p and *THY1* respectively. A dissolution curve was referred to for the evaluation of the reliability of the obtained PCR results. Cycle threshold (*C*_t_) value was selected and used as the inflection point on the amplification power curve, Δ*C*_t_ = *C*_T_ (target gene) − *C*_T_ (internal control), ΔΔ*C*_t_ = Δ*C*_t_ (the experimental group) − Δ*C*_t_ (the control group). The relative expression of target gene was calculated using the formula 2^−ΔΔ*C*_t_^ [23]. All experiments were repeated three times in an independent fashion.

**Table 1:** Primer sequences for RT-qPCR

Gene		Sequences (5′–3′)
*miR-140-5p*	RT Primer	CAGTGCAGGGTCCGAGGTCAGAGCCACCTGGGCAATTTTTTTTTTTCTACCA
*U6*	RT Primer	GTCGTATCCAGTGCAGGGTCCGAGGTATTCGCACTGGATACGACAAAATATGGAAC
*miR-140-5p*	Forward	ACACTCCAGCTGGGCAGTGGTTTTACCCTA
	Reverse	TGGTGTCGTGGAGTCG
*U6*	Forward	TGCGGGTGCTCGCTTCGGCAGC
	Reverse	CCAGTG CAGGGTCCGAGGT
*THY1*	Forward	CAGGACGGAGCTATTGGCACCAT
	Reverse	ACGGCAGTCCAGTCGAAGGTTCT
*GAPDH*	Forward	TGAAGGTCGGAGTCAACGGATTTGGT
	Reverse	CATGTGGGCCATGAGGTCCACCAC

### Western blot analysis

Total protein was extracted from both the tissues and cells, and the concentration was determined according to the instructions on the bicinchoninic acid (BCA) kit (Boster Biological Technology., Ltd, Wuhan, Hubei, China). The protein was then mixed with the loading buffer (30 µg/well) and heated at 95°C for 10 min. Ten percent polyacrylamide gel electrophoresis (PAGE) (Boster Biological Technology., Ltd, Wuhan, Hubei, China) was employed in order to separate the proteins at electrophoresis voltages from 80 to 120 V, with the wet transfer method used at 100 mV transmembrane voltage for 45–70 min. The protein was transferred on to a polyvinylidene fluoride (PVDF) membrane, followed by blockade using 5% bovine serum albumin (BSA) for 1 h at room temperature. The membrane was then probed with the diluted (1:1000) primary antibodies to *THY1* (ab92574), caspase-3 (ab32042), Bcl-2 associated X protein (Bax) (ab32503), B-cell lymphoma-2 (Bcl-2) (ab59348), cleaved poly(ADP-ribose) polymerase 1 (PARP1) (ab32064), Notch 1 intracellular domain (NICD) (ab8925), hairy-related protein (H)ES)1, (ab71559), HES5 (ab25374), E-cadherin (ab15148), vimentin (ab137321), N-cadherin (ab18203), matrix metalloproteinase (MMP)-2 (ab37150), MMP-9 (ab38898), β-actin (ab8226) at 4°C overnight. All antibodies were purchased from Abcam (Cambridge, MA, U.S.A.). The membrane was rinsed three times using the Tris-buffered saline tween (TBST; 5 min each), followed by an incubation with horseradish peroxidase (HRP)-labeled secondary antibody for 1 h. The membrane was washed three times with TBST (5 min each). β-actin was regarded as the internal reference. According to instructions of the SuperSignal® West Dura Extended Duration Substrate, approximately 1 ml enhanced chemiluminescence (ECL) was prepared, which was incubated with the membranes for 1 min, followed by the removal of the excess ECL agent. The protein bands were developed after exposing the X-ray film for 5–10 min and photographed by Bio-Rad Gel Dol EZ (GEL DOC EZ IMAGER, Bio-Rad, Hercules, CA, U.S.A.). ImageJ software was applied for analysis of the gray value of the target band. Each experiment was performed in triplicate.

### 3-(4,5-dimethylthiazol-2-yl)-5(3-carboxymethonyphenol)-2-(4-sulfophenyl)-2H-tetrazolium assay

GC cells in logarithmic growth phase of each transfection group were seeded in a 96-well plate at a density of 5 × 10^3^ cells per well (100 μl each well). The cells were cultured in a CO_2_ incubator for 24, 48, and 72 h respectively at 37°C. Afterward, 20 μl MTS (3-(4,5-dimethylthiazol-2-yl)-5(3-carboxymethonyphenol)-2-(4-sulfophenyl)-2H-tetrazolium) reagent (G3582, Promega Corporation, Madison, WI, U.S.A.) was added in each well and incubated for another 4 h. The optical density (OD) of each well was measured at a wavelength of 490 nm using a microplate reader (SpectraMax M5, Molecular Devices, San Jose, CA, U.S.A.). The GC cell survival rates were calculated using the following formula: cell survival rate (%) = OD value of the experimental group/OD value of the control group × 100%. All experiments were repeated in triplicate.

### Wound-healing assay

The GC cells were seeded in a six-well plate and transfected, followed by an incubation at 37°C until cells adhered to the well. A line was drawn in the middle of well using a sterilized pipette tip in order to examine GC cell migration. The scratch area was photographed and the same vision in the well was marked for convenience location purposes for the following occasion. The timing point was set as the 0th h. The cell culture medium was removed after an incubation for 24 h at 37°C. The plate was washed three times with PBS to remove the cellular debris from wound-healing, after which serum-free medium was added. Photographs were subsequently obtained using an Olympus inverted microscope (Olympus Optical Co., Ltd., Tokyo, Japan) and the timing point was set as the 24th h. Six fixed vision fields were selected and a click-counting software was used to calculate the cell number in the scratching areas. All experiments were repeated in triplicate.

### Transwell assay

A total of 60–80 μl Matrigel (3.9 mg/ml) was added into the Transwell chamber (140629, Thermo Fisher Scientific Inc., Waltham, MA, U.S.A.) and incubated for 30 min at 37°C until the Matrigel was solidified. The pre-warmed culture medium was added to the plate, which was then placed in the incubator at 37°C for a 2-h hydration. Transwell chamber was placed in each well and added with 0.5 ml cell suspension (5 × 10^4^ cells/ml) for 24 h at 37°C. Afterward, the cells on the apical chamber were washed with PBS. The cells in the basolateral chamber were fixed with pre-cooled methanol for 30 min and stained with 0.1% Crystal Violet solution for 10 min. The cells were photographed under an Olympus inverted microscope. Six visions with fixed positions were selected and the migratory cells to the basolateral chamber were calculated using the click-counting software. All experiments were repeated in triplicate.

### Flow cytometry

After a 24-h period of transfection, the cells were collected and washed with cold PBS. The cell precipitation was resuspended with PBS containing calcium into cell suspension at a density of 1 × 10^6^ cells/ml. A volume of 100 µl cell suspension was placed in a tube at room temperature and mixed with 10 mg/ml propidium iodide (PI, P4170, Sigma–Aldrich Chemical Company, St. Louis, MO, U.S.A.) and 10 mg/ml RNase A. The mixture was incubated at 4°C for 30 min followed by the addition of 400 µl staining buffer. Flow cytometer (BD Bioscience, San Diego, CA, U.S.A.) was utilized in order to analyze a total of 10^4^ cells. Cell Quest software was employed for data analysis. Annexin V^+^ cells were identified as apoptotic cells, while PI^+^ Annexin V^−^ cells were necrotic cells. The apoptosis rate was calculated using the formula: Apoptosis rate = (Annexin V^+^PI^+^ cell numbers + Annexin V^+^PI^−^cell numbers)/10^4^ × 100%). All experiments were repeated in triplicate.

### Statistical analysis

All experiments were conducted in triplicate. SPSS21.0 software (IBM Corp. Armonk, NY, U.S.A.) was applied for analysis of the data and the mean and standard deviation (SD) were calculated. Measurement data were presented as mean ± SD. The difference between two groups was analyzed using a *t* test, while one-way analysis of variance (ANOVA) was applied for comparing among multiple groups. Homogeneity of variance was conducted using variance analysis, while heterogeneity of variance was conducted using the Wilcoxon’s rank sum test. The correlations between gene expression and clinical case were analyzed by the Chi-square test and Fisher’s exact test. A value *P*<0.05 was considered to be statistically significant.

## Results

### Microarray-based gene expression profiling of GC

In order to ascertain whether miR-140-5p influences GC by regulating *THY1* and the Notch signaling pathway, screening of the differentially expressed genes from the GC-related datasets was performed. The GEO database was employed to screen the GC-related datasets, hence GSE13861, GSE65801 and GSE79973 were obtained. Following the analysis of the differentially expressed genes in the GC samples and normal samples in these three datasets, 132, 520 and 329 differentially expressed genes were subsequently obtained from the three datasets respectively. Figure 1A–C depicts the heatmaps of the top 100 differentially expressed genes. A Venn analysis was used to screen genes related to GC, and the intersections of the differentially expression genes in the three datasets were obtained, with nine differentially expressed genes determined (Figure 1D). The MalaCards database was used to select GC-related genes, from which ten genes including TP53, and ERBB2 were selected. Association analysis among the nine differentially expressed genes and GC-related genes was conducted, and a network map of gene interaction was constructed (Figure 1E). The results obtained revealed that the ATP4A and *THY1* genes were located in a more central position in relation to the nine differentially expressed genes, with the functions of the two aforementioned genes subsequently obtained. Multiple studies have been performed aiming to identify the mechanism of ATP4A in GC [24,25]. However, a relatively scarce amount of literature exists regarding *THY1*. Hence, *THY1* was selected as the main target of the present study. Existing studies have demonstrated the close correlation of *THY1* gene with the Notch signaling pathway [26,27], with some even claiming the involvement of the Notch signaling pathway in GC [28,29]. On the basis of these studies, our team of researchers hypothesized the participation of *THY1* in GC by mediating the Notch signaling pathway. The mirDIP database and miRGator database were employed to predict miRs that regulated *THY1* in order to thoroughly demonstrate the upstream regulation mechanism of *THY1* gene. There were 12 regulating miRs in the mirDIP database and 373 regulating mRNAs in the miRGator database. Figure 1F represents the intersection of the top 150 miR from the mirDIP database prediction results and the miRGator database prediction results, and four miRs were selected in the intersection. Certain studies have highlighted the poor expression of miR-140-5p in GC, suggesting that miR-140-5p could repress GC development [30,31]. Taken together, we subsequently asserted that miR-140-5p could participate in GC by regulating the *THY1-*dependent Notch signaling pathway.

**Figure 1:** *THY1* and miR-140-5p are engaged in the progression of GC (**A**–**C**) Heatmaps of differentially expressed genes. The transversal coordinates represent the sample number, the ordinate represents the name of the gene, the left dendrogram represents the gene expression clustering, and each small square in the graph is the level of a gene in one sample. The histogram of the upper right is the color order. (**D**) Venn analysis of the top 100 differentially expressed genes in three datasets, and the center area represents the intersection of three datasets. (**E**) Interaction analysis between differentially expressed genes and GC-related genes, each cycle stands for a gene and the line between cycles indicates the interaction between genes. The brighter the color of the circle indicates that the gene is at the core in the network map. The red font represents the GC-related genes obtained in the MalaCards database, and the black font represents the differentially expressed gene in GC. (**F**) The prediction results of the regulatory miRs of *THY1*, the left cycle is the prediction results of the mirDIP database, the right cycle indicates the top 150 miRs of the miRGator database, and the middle part indicated the intersection of the prediction results of the two datasets.

### Lower expression of miR-140-5p and higher expression of *THY1* in GC tissues

Following our speculation in regard to whether miR-140-5p had the potential to affect GC by regulating *THY1*, the attention and focus in the experiment shifted to identify the expression of miR-140-5p and *THY1* in GC tissues and the paracancerous tissues. A difference was observed in the miR-140-5p and *THY1* expression between the GC tissues and the paracancerous tissues, based on the results of RT-qPCR and Western blot analysis (Figure 2A–D). A correlation investigation into miR-140-5p and the expression of *THY1* among the GC tissue samples was performed, which revealed that miR-140-5p was negatively correlated with *THT1* (Figure 2E). These results provided conclusive evidence suggesting revealing there to be lower expression of miR-140-5p in GC tissues compared with the paracancerous tissues, in contrast with higher expression of *THY1*.

**Figure 2:** miR-140-5p is poorly expressed and *THY1* is overexpressed in GC tissues (**A**) Expression of miR-140-5p in GC tissues and paracancerous tissues detected by RT-qPCR. (**B**) mRNA expression of *THY1* in GC tissues and paracancerous tissues detected by RT-qPCR. (**C**) Protein bands of THY1 in GC tissues and paracancerous tissues detected by Western blot analysis. (**D**) Quantitative analysis of THY1 protein expression in GC and paracancerous tissues. (**E**) Correlation analysis of miR-140-5p expression and the mRNA expression of *THY1* in GC and paracancerous tissues; *, *P*<0.05.

### The expression of miR-140-5p and *THY1* is correlated to the progression of GC

The next experiment was based on analyzing the relationship between miR-140-5p and *THY1* expression and the clinicopathological characteristics in GC. The clinicopathological characteristics of all GC patients were analyzed and organized accordingly. According to the median levels of miR-140-5p and *THY1*, GC patients were classified into low and high expression groups [30]. The results revealed that there was no existence of a correlation between the miR-140-5p expression and gender and age, whereas a significant correlation was observed with differentiation degree (*P*=0.026), lymph node metastasis (*P*=0.002), clinical stage (*P*=0.033) and infiltration degree (*P*=0.018) of GC patients. Similarly, no associations were observed between the expression of *THY1* and gender and age, whereas significant correlations existed with differentiation degree (*P*<0.001), lymph node metastasis (*P*<0.001), clinical stage (*P*=0.003) and infiltration degree (*P*=0.001) of GC patients (Table 2).

**Table 2:** The relationship between miR-140-5p and THY1 and clinicopathological characteristics of GC

Factor	Case	miR-140-5p high expression	miR-140-5p low expression	*P*	*THY1* high expression	*THY1* low expression	*P*
Age (years)				0.555			0.844
≤55	42	24	18		23	19	
>55	63	32	31		33	30	
Gender				0.544			0.104
Male	67	34	33		40	27	
Female	38	22	16		16	22	
Differentiation				0.026			<0.001
Well	27	10	17		23	4	
Moderate	34	16	18		18	16	
Poor	44	30	14		15	29	
Lymph node metastasis				0.002			<0.001
Yes	60	24	36		42	18	
No	45	32	13		14	31	
Clinical stage				0.033			0.003
I	9	7	2		3	6	
II	18	14	4		4	14	
III	47	21	26		26	21	
IV	31	14	17		23	8	
Infiltration degree				0.018			0.001
Serosal invasion	59	25	34		40	19	
Without serosal invasion	46	31	15		16	30	

### SGC-7901 and MGC-803 cell lines are selected for subsequent experiments

The expression of miR-140-5p and *THY1* in the normal gastric epithelial cell line (GES-1) and GC cell lines (MKN-28, MGC-803, SGC-7901, AGS and MKN-45) were detected (Figure 3). The expression of miR-140-5p in GES-1 was notably higher than the GC cell lines, while SGC-7901 exhibited the lowest miR-140-5p expression. An opposite trend was observed in regard to the relative expression trend of *THY1* in all cell lines compared with the expression of miR-140-5p, which was lowest in GES-1 and highest in SGC-7901 (all *P*<0.05). Based on the above results, the GC cell line SGC-7901 was selected for subsequent experiments, and GC cell line MGC-803 was employed in the process of verifying the results.

**Figure 3:** SGC-7901 and MGC-803 cell lines are selected for subsequent experiments (**A**) miR-140-5p expression measured by RT-qPCR. (**B**) mRNA expression of *THY1* measured by RT-qPCR. (**C,D**) Protein expression of THY1 detected by Western blot analysis; *, *P*<0.05.

### *THY1* is a target of miR-140-5p

The targeting relationship between miR-140-5p and *THY1* was determined by means of bioinformatics prediction and determination of luciferase activity. The online bioinformatics software at microrna.org predicted *THY1* as the downstream target gene of miR-140-5p (Figure 4A). The result revealed there to be a significant decrease in luciferase activity in the miR-140-5p mimic and *THY1*-wt groups in contrast with the NC + *THY1*-wt group (Figure 4B). These findings indicated that *THY1* was indeed a target gene of miR-140-5p.

**Figure 4:** miR-140-5p specifically binds to *THY1* (**A**) Binding sites of miR-140-5p and *THY1* predicted by the online bioinformatics software, microrna.org. (**B**) Dual-luciferase reporter gene assay for confirmation of the targeting relationship between miR-140-5p and *THY1*; *, *P*<0.05 *vs*. the NC + *THY1*-wt group. The wt sequence of *THY1* was 5′-CCUGACUUCUCCCCAA***CCA***CUU-3′ and mut sequence was 5′-CCUGACUUCUCCCCAA***UUG***CUU-3′.

### miR-140-5p overexpression suppresses *THY1* expression and the activation of the Notch signaling pathway

This segment of the experiment placed an emphasis on determining the mechanism by which miR-140-5p influences the Notch signaling pathway via *THY1*. The expression of miR-140-5p, *THY1* and Notch signaling pathway-related proteins NICD, HES1 and HES5 in SGC-7901 cells after transfection were determined by RT-qPCR and Western blot analysis. On the basis of these results, it was concluded that an increase in miR-140-5p expression along with a decrease in *THY1* and *Notch1* could result in the significant reductions in the expression of *THY1* and Notch signaling pathway-related proteins NICD, HES1 and HES5. The decrease in miR-140-5p expression could remarkably induce the expression of *THY1* and Notch signaling pathway-related proteins NICD, HES1 and HES5. Contrarily, si-*THY1* and si-*Notch1* could reverse the promotive effects miR-140-5p inhibitor exerted on the expression of Notch signaling pathway-related proteins NICD, HES1 and HES5 (all *P*<0.05; Figure 5). These were consistent with the results that displayed by GC cell line MGC-803 (Supplementary Figure S1). The above results revealed that miR-140-5p suppresses the activation of the Notch signaling pathway.

**Figure 5:** miR-140-5p negatively regulates the expression of proteins in the Notch signaling pathway in SGC-7901 cells (**A**) Expression of miR-140-5p in SGC-7901 cells after transfection detected by RT-qPCR. (**B**) mRNA expression of *THY1* in SGC-7901 cells after transfection detected by RT-qPCR. (**C**) Protein expression of *THY1* in SGC-7901 cells after transfection detected by Western blot analysis. (**D**) Gray value analysis of *THY1* protein. (**E**) Expression of Notch signaling pathway-related proteins (NICD, HES1, HES5). (**F**) Gray value analysis of Notch signaling pathway-related proteins (NICD, HES1, HES5); *, *P*<0.05 *vs*. the control group, ^#^, *P*<0.05 *vs*. the NC group; ^&^, *P*<0.05 *vs*. the si-NC group; ^∆^, *P*<0.05 *vs*. the miR-140-5p inhibitor group.

### miR-140-5p overexpression inhibits proliferation of GC cells

Based on the data research findings which revealed that miR-140-5p was poorly expressed and THY1 was highly expressed in GC cell line SGC-7901, the objective of the subsequent experiment was moved to identify the role of miR-140-5p in the biological process of cell proliferation. The proliferation of the transfected SGC-7901 cells was investigated using MTS assay. The SGC-7901 cell proliferation was decreased after the cells were transfected with miR-140-5p mimic, si-*THY1* or si-*Notch*. miR-140-5p inhibitor + si-*THY1* and miR-140-5p inhibitor + si-*Notch1* could significantly reverse the promotion of SGC-7901 cell proliferation induced by miR-140-5p inhibitor (all *P*<0.05; Figure 6). These were consistent with the results displayed by GC cell line MGC-803 (Supplementary Figure S2). These results concluded that miR-140-5p overexpression inhibited the proliferation of GC cells.

**Figure 6:** miR-140-5p overexpression inhibits proliferation of SGC-7901 cells *, *P*<0.05 *vs*. the control group.

### miR-140-5p overexpression suppresses migration and invasion of GC cells

The effects of miR-140-5p on the migration and invasion of transfected SGC-7901 cells were examined by wound-healing and Transwell assays (Figure 7). Cell migration and invasion were distinctly suppressed by miR-140-5p mimic, si-*THY1* and si-*Notch1*. A key observation revealed that miR-140-5p inhibitor could reverse the inhibitory effect. However, upon silencing the expression of *THY1* gene and Notch, no significant effect was noted from the miR-140-5p inhibitor on the migration and invasion of SGC-7901 cells (all *P*<0.05). N-cadherin, vimentin, MMP-2, MMP-9 expression in SGC-7901 cells was significantly inhibited, and E-cadherin was enhanced after treatment with miR-140-5p mimic, si-*THY1* and si-*Notch1*. The miR-140-5p inhibitor stimulated the expression of N-cadherin, vimentin, MMP-2 and MMP-9 in SGC-7901 cells, whereas inhibited the expression of E-cadherin. The results indicated that si-*THY1* and si-*Notch1* can reverse the promotion of N-cadherin, vimentin, MMP-2, MMP-9 expression in SGC-7901 cells and the inhibition of E-cadherin expression by miR-140-5p inhibitor. All of which were identical with the results that displayed by GC cell line MGC-803 (Supplementary Figure S3). Thus, we concluded that miR-140-5p suppressed the migration and invasion of GC cells.

**Figure 7:** miR-140-5p overexpression leads to the suppression of migration and invasion of SGC-7901 cells (**A**) SGC-7901 cell migration detected by wound-healing. (**B**) SGC-7901 cell invasion detected by Transwell assay. (**C**) Statistical analysis of (A). (**D**) Statistical analysis of (B). (**E**) Expression of *N-cadherin, vimentin, MMP-2, MMP-9, E-cadherin* in SGC-7901 cells after transfection detected by RT-qPCR; *, *P*<0.05 *vs*. the control group; ^#^, *P*<0.05 *vs*. the NC group; ^&^, *P*<0.05 *vs*. the si-NC group; ^∆^, *P*<0.05 *vs*. the miR-140-5p inhibitor group.

### miR-140-5p overexpression promotes apoptosis of GC cells

Flow cytometry assay was adopted to detect the effects of miR-140-5p on apoptosis of SGC-7901 cells. The number of apoptotic cells were higher in the miR-140-5p mimic group, the si-*THY1* and si-*Notch1* groups compared with the control and NC groups. In contrast with the control and si-NC groups, a significant decrease was detected regarding the cell apoptosis in the miR-140-5p inhibitor group. The cell apoptosis of the miR-140-5p inhibitor + si-*THY1* group and the miR-140-5p inhibitor + si-*Notch1* group was obviously increased when compared with the miR-140-5p inhibitor group (all *P*<0.05) (Figure 8A,B). These were in accord with the findings based on the GC cell line MGC-803 observations (Supplementary Figure S4), which ultimately indicated that miR-140-5p promoted the apoptosis of GC cells.

**Figure 8:** miR-140-5p overexpression promotes apoptosis of SGC-7901 cells (**A**) Apoptosis of SGC-7901 cells in each group by flow cytometry. (**B**) Histogram of apoptosis of each group; *, *P*<0.05 *vs*. the control group; ^#^, *P*<0.05 *vs*. the NC group; ^&^, *P*<0.05 *vs*. the si-NC group; ^∆^, *P*<0.05 *vs*. miR-140-5p inhibitor group.

### miR-140-5p overexpression promotes expression of pro-apoptotic protein and suppresses anti-apoptotic protein

The role of miR-140-5p in regulating the expression of apoptosis-related proteins was investigated. The expression of the activated caspase-3, Bax, Bcl-2 and cleaved PARP1 was examined through the application of Western blot analysis, with the relative levels calculated normalized to the gray value of β-actin (Figure 9A–D). Compared with the control and NC groups, SGC-7901 cells delivered with miR-140-5p mimic displayed a significantly higher expression of activated caspase-3, Bax and cleaved PARP1, and decreased expression of Bcl-2. However, treatment with miR-140-5p inhibitor in SGC-7901 cells resulted in a diminished expression of activated caspase-3, Bax and cleaved PARP1, along with a higher expression of Bcl-2. In comparison with the si-NC and control groups, the activated caspase-3, Bax and cleaved PARP1 expression increased, whereas the Bcl-2 expression decreased in the si-*THY1* and si-*Notch1* groups. Compared with the miR-140-5p inhibitor group, an increased expression of activated caspase-3, Bax and cleaved PARP1 was observed, whereas a decreased Bcl-2 expression was found in the miR-140-5p inhibitor + si-*THY1* group and the miR-140-5p inhibitor + si-*Notch1* group (all *P*<0.05). Consistent findings were detected by the GC cell line MGC-803 (Supplementary Figure S5). These findings strongly indicated that miR-140-5p, by negative regulating *THY1*, blocked the activation of Notch signaling pathway, thus increasing the expression of pro-apoptotic protein and decreasing the expression of anti-apoptotic protein.

**Figure 9:** miR-140-5p overexpression promotes expression of pro-apoptotic protein and suppresses expression of anti-apoptotic protein in SGC-7901 cells (**A**) Apoptosis-related proteins expression in SGC-7901 cells detected by Western blot analysis. (**B**) Statistical analysis of (A). (**C**) The protein expression of cleaved PARP1 detected by Western blot analysis. (**D**) Statistical analysis of (C). *, *P*<0.05 *vs*. the control group; ^#^, *P*<0.05 *vs*. the NC group; ^&^, *P*<0.05 *vs*. the si-NC group; ^∆^, *P*<0.05 *vs*. the miR-140-5p inhibitor group.

## Discussion

Various studies have provided evidence elucidating the role and mechanism by which various miRs act to regulate various tumor-related genes along with their carcinogenic influence in GC [32,33]. The current study aimed to identify whether miR-140-5p influences GC and the mechanism and involvement of the *THY1*-dependent Notch signaling pathway. Our findings demonstrated that miR-140-5p inhibited cell proliferation, migration, and invasion through negative regulation of Notch signaling pathway via *THY1* in GC.

The biological function of miR-140 has only been investigated in a limited number of malignant carcinomas including breast cancer, osteosarcoma, colon cancer, hepatocellular carcinoma and non-small cell lung cancer [34–37]. Studies have highlighted the various roles played by miR-140 in regulating tumor cell phenotype, for example, miR-140 inhibits the self-renewal and growth of breast cancer stem cells [38], and dampens the invasion of esophageal cancer cells [39]. A key finding suggested the frequent occurrence of an aberrant expression of miR-140-5p in various cancers, which placed further emphasis on the significance of the influence of miR-140-5p on the initiation and progression of tumors [12]. A recent study found that miR-140 was significantly reduced in colorectal cancer tissues, and its down-regulation was associated with advanced tumor node metastasis stage and distant metastasis of colorectal cancer, and suggested that miR-140 overexpression inhibits the cell migration and invasion of colorectal cancer [40]. The results of the current study revealed there to be a decreased expression of miR-140-5p in GC patients, while further indicating that miR-140-5p up-regulation inhibited the migration, invasion and proliferation, and promoted the apoptosis of GC. As a recent study revealed, upon overexpression of miR-140-5p, that the protein levels of vimentin, MMP2 and MMP3 were all significantly reduced, while the protein level of E-cadherin was remarkably enhanced in GC cells, which ultimately resulted in the inhibition of GC cell proliferation, migration and invasion [30].

The results obtained from the current study demonstrated distinctly higher expression of *THY1* in GC in comparison with that of adjacent tissues according to RT-qPCR and Western blot analysis. *THY1* is a multifunctional signaling modulator that plays a role in the processes of cell adhesion, proliferation, survival, cytokines and growth factors [41]. *THY1* is defined as a tumor stem cell markern GC, lung cancer, esophageal cancer and hepatocellular carcinoma; due to its participation in various cellular processes [42]. During the *in vivo* differentiation and anti-chemotherapy, self-renewal ability was noted to be enhanced, while tumor development was induced in the CD90^+^ (*THY1*) positive tumor initiating cell population [43]. The expression of *THY1* is up-regulated in GC tissues, where it could potentially inhibit the apoptosis of GC cells by regulating the level of SPARC protein, and CD90^+^(*THY1*) cells that have a greater potential to initiate tumor formation as well as the process of self-renewal *in vivo* [11]. The expression of *Notch1* in GC tissues was significantly higher compared with the normal gastric tissues, and is critical in the mediation of tumor size and differentiation, infiltration and depth of blood vessel invasion [44]. Previous studies have suggested that the *Notch1* and Notch2 signaling pathways are activated in GC cells, while studies have speculated regarding the involvement of the Notch signaling pathway in tumor formation and development, suggesting the Notch signaling pathway is implicated in tumorigenesis [20]. The Notch family proteins play a crucial functional role in mediating cell proliferation, differentiation and apoptosis [45]. Brzozowa et al. [46] provided evidence highlighting a correlation between the Notch signaling pathway and the pathogenesis of gastrointestinal tumors including gastric and colon cancers. On the basis of this evidence, *Notch1* due to its abilities could potentially be used as a prognostic indicator for GC [47]. Besides, a former study also concluded that *Notch1* silencing could reduce the anti-apoptotic protein Bcl-2, and increase the concentration of the pro-apoptotic protein Bax [48], while the current study observed that GC cells introduced with miR-140-5p inhibitor as well as si-*Notch* exhibited increased activated caspase-3, Bax and cleaved PARP1, along with decreased Bcl-2.

In addition, *THY1* was found to be a target gene of miR-140-5p. The up-regulation of miR-140-5p leads to a diminished expression of *THY1* as well as inactivated Notch signaling pathway. Furthermore, miR-140-5p was found to be negatively correlated with *THY1* in the GC tissue samples*.* The regulation of the Notch signaling pathway by specific miRs has been suggested as a novel therapy for GC treatment [29]. Studies have demonstrated that miR-140-5p is involved in the inhibition of tumor invasion and metastasis by suppressing the activity of the disintegrin-like metalloproteinase10 (ADAM10)-mediated Notch signaling pathway, and a decrease in the Notch signaling pathway would consequently inhibit the invasion and migration of FaDu cells, thereby highlighting the vitality of miR-140-5p in the inhibition of FaDu cells [14]. Moreover, consistent findings from a previous study revealed that overexpression of miR-124 resulted in decreased levels of Notch signaling pathway related proteins (NICD, HES1 and HES5), GC cell invasion, migration, and proliferation, in addition to increased apoptosis rate [29].

## Conclusion

In conclusion, the current study presents evidence highlighting the ability of miR-140-5p to reduce migration, invasion and proliferation, and accelerate the apoptosis of GC cells through suppression of *THY1* and inactivation of the Notch signaling pathway. The up-regulation of miR-140-5p plays a positive role in suppressing the development of GC cells (Figure 10). Our study offers further insight into the underlying molecular mechanism of miR-140-5p in the development of GC. However, due to limited experimental conditions, further investigations into the molecular mechanisms of miR-140-5p–based GC therapeutic strategies are required.

**Figure 10:** miR-140-5p participates in GC cell proliferation, migration, invasion and apoptosis by mediating Notch signaling pathway via *THY1* miR-140-5p is poorly expressed in GC and *THY1* is overexpressed in GC. miR-140-5p down-regulates *THY1* expression. *THY1* gene activates the Notch signaling pathway, and results in the inhibition of caspase-3 and Bax expression and promotes the expression of Bcl-2, which ultimately affects the proliferation, migration, invasion and apoptosis of GC.

## Supporting information

**Supplementary Figure S1:** 

**Supplementary Figure S2:** 

**Supplementary Figure S3:** 

**Supplementary Figure S4:** 

**Supplementary Figure S5:** 

## Abbreviations

ADAM10: disintegrin-like metalloproteinnase10
Bax: Bcl-2 Associated X Protein
*C*_t_: cycle threshold
ECL: enhanced chemiluminescence
FBS: fetal bovine serum
GC: gastric cancer
GEO: Gene Expression Omnibus
GES-1: gastric epithelial cell
miR: microRNA
miR-140-5p: microRNA-140-5p
MMP: matrix metalloproteinase
MTS: 3-(4,5-dimethylthiazol-2-yl)-5(3-carboxymethonyphenol)-2-(4-sulfophenyl)-2H-tetrazolium
NC: negative control
NICD: Notch1 intracellular domain
OD: optical density
PAPR1: poly(ADP-ribose) polymerase 1
PI: propidium iodide
RT-qPCR: reverse-transcription quantitative polymerase chain reaction
SD: standard deviation
SPARC: Secreted Protein Acidicand Rich in Cysteine
TBST: Tris-buffered saline tween
THY1: thymus cell antigen 1
THY1-mut: *THY1*-3′-UTR-mut
THY1-wt: *THY1*-3′-UTR-wt
UTR: untranslated region
U6: small nuclear RNA U6
wt: wild-type
